# Evaluation of Application Effect of Self-Made Compression Cold Therapy in Postoperative Rehabilitation of Patients with Orthopedic Dyskinesia

**DOI:** 10.1155/2022/8222933

**Published:** 2022-07-18

**Authors:** Xiaojuan Wan, Liping Ji, Min Zhao, Shixiang Zhu, Meixiu Tang

**Affiliations:** The People's Hospital of Rugao, Nantong, Jiangsu 226500, China

## Abstract

With the accelerated aging of the population, orthopedic injuries have become more collective. Among them, the incidence of ankle fractures remains high. Surgery is an effective way to treat ankle fractures by utilizing special surgical site, complex anatomical structure, and specific surgical methods. With surgical approach, it is easy for basis postoperative blood loss, pain, swelling, and other problems. After surgery, most patients suffer from symptoms of fear, increased pain sensitivity, and excessive irrational concerns about physical movement or activity. Compression cold therapy combines cold therapy with air pressure therapy to ease local exudation, constrict blood vessels, improve circulation, relieve pain, and control inflammation through the effects of low temperature and pressure. Application during the rehabilitation period can prevent joint swelling, reduce muscle soreness, and promote the functional recovery of limbs, which provides an effective guarantee for postoperative rehabilitation of patients with orthopedic dyskinesia. Based on this, it is very important to evaluate the application and effect of self-made compression cold therapy in postoperative rehabilitation of patients with orthopedic dyskinesia. This work proposes a one-dimensional deep convolutional neural network-based method; DenseNet for analyzing the rehabilitation effect of patients with orthopedic dyskinesia after ankle fracture surgery. The approach is to evaluate the rehabilitation effect of self-made compression cold therapy from the perspectives of feature reuse, attention mechanism, and feature decoupling. Experiments on the dataset show that the proposed neural network has better efficacy evaluation performance. The proposed systematic assessment based on the emerging deep learning network has great significance in healthcare domain, particularly in assessing applicability, side effects, and noninvasiveness of treatment methods.

## 1. Introduction

The ankle joint, also known as the talus calf joint, is one of the most important joints in the human body that plays an irreplaceable role in daily life and sports. The ankle joint connects the lower end of tibia and the lower end of the fibula. The talus constitutes the bony structure of the ankle joint. The lower end of the tibia and fibula shapes the articular surface of the talus. The medial malleolus articular surface, the lateral malleolus articular surface, the articular surface of the lower end of the tibia, and the posterior malleolus constitute the ankle point, which accommodates the talus joint head. The wider anterior part of the joint head enters the socket when the foot is dorsiflexed, and the joint is stabilized. However, in plantar flexion, the narrower posterior part enters the socket, and the ankle joint loosens at this time and is prone to sprain. As overt from the anatomical structure of the ankle joint, the lateral malleolus is lower than the medial malleolus on the coronal plane, and the lateral malleolus is more posterior than the medial malleolus on the sagittal plane. This limits retroversion of the talus, so ankle injuries are most collective in the varus [1]. The stress area of the ankle joint is smaller than that of the knee and hip joint and is the weight-bearing joint closest to the ground [2–6].

Enhanced recovery after surgery (ERAS), which has been advocated in recent years, refers to the implementation of various proven and effective methods through the perioperative period. It further reduces the traumatic stress of surgical patients, reduces the incidence of various complications, and achieves the purpose of reducing the mortality rate and shortening the length of hospital stay. This speeds up the patient's recovery, where effective analgesia and early postoperative mobilization are important elements of accelerated recovery. In the early stage of fracture injury, the body releases inflammatory response factors, proteases, and other substances, which increase the permeability of local blood vessels. This causes varying degrees of swelling and pain in the joints, and in severe cases, skin tension blisters, which affect the course of surgical treatment and increase the risk of infection. Postoperative swelling and pain are mostly related to surgical incision and intraoperative tissue damage. In severe cases, it will affect the functional exercise and rehabilitation process of the patient's joints. This prolongs the patient's bed rest time and increases the risk of lower extremity venous thrombosis and other complications. The ankle joint is an important joint for people's daily activities and walking. After the injury, normal life and work of the patients will be affected. If the treatment and rehabilitation are not warranted timely, it may also lead to long-term physical and psychological problems [7–11].

Cold therapy induces effects at the application site and spinal cord level through neural and vascular mechanisms, reducing the activation threshold of tissue nociceptors and the velocity of pain nerve signaling. Current research illustrations show that cold therapy reduces tissue blood flow, lowers the temperature of the superficial skin and subcutaneous tissue, slows cell metabolism, and inhibits cell activity [12]. A bone scan study found that 20 minutes of ice on one knee reduced arterial blood flow by 38% and soft tissue blood flow by 26% [13]. Bone resorption, which reflects changes in bone blood flow and metabolism, was reduced by 19%. The traditional ice treatment effect is not ideal, and there are disadvantages such as difficult temperature control, poor patient experience, and easy occurrence of frostbite. At room temperature, condensation droplets that form on the surface of the ice pack may contaminate the cut. The self-made pressure cold therapy device combines cold therapy with pressure therapy and has the advantages of soft material, large coverage area, stable temperature, and pressure, etc. At present, it has been widely used in the rehabilitation of soft tissue injury, joint replacement perioperative period, and fracture patients and has achieved good clinical results [14–17]. The recent approaches proposed in [18–20] may be helpful in predicting and evaluating the therapeutic effect and ensuring accurate decision making [21] in the realm of orthopedics.

Usually, surgery is advised to the patients suffering from kinesiophobia. Therefore, it becomes pertinent to evaluate the therapeutic effect of the self-compressed cold therapy device on patients after orthopedic surgery, which will help to formulate more appropriate rehabilitation measures. The neural network is the evolving machine learning method that can be rightly used in the systematic evaluation. This work utilizes neural networks in the medical domain and proposes a method for evaluating the therapeutic effect of self-made compression cold therapy on patients with dyskinesia. By comparing outcomes of the approach with the contemporary methods, it is revealed that the proposed 1D-DenseNet is more robust and accurate. Unlike other convolution neural networks, the approach of separable convolution is applied to the dense module. Moreover, to reduce feature map, an average pooling layer is used in the transition module. A comparatively promising information flow is obtained by escaping residual connections and utilizing fewer parameters. With 96.7% precision and 93.9% recall, an improved 3.2% precision was achieved. The approach recommended has great significance in physical and occupational therapy particularly in assessing applicability of treatment methods followed for cerebral palsy and joint contractures disorders.

The paper arrangements are as follows: Section 2 discusses the related work.  Section 3 evaluates the various methods.  Section 4 analyzes the experiment and discussion.  Section 5 concludes the article.

## 2. Related Work

Leyes et al. [22] mentioned that the incidence of complications after ankle fracture is 5% to 40%, which may occur during conservative treatment and surgical treatment. It is stated in [23] that pain and swelling often occur in the early stage of injury, which causes inconvenience to patients' daily life and exercise, and also increases the medical burden on society. Vuurberg et al. [24] mentioned that the ankle joint is mostly wrapped by blood vessels and tendons. Affected by gravity and the immobilization of the affected limb, the venous and lymphatic drainage of the lower extremity is not smooth, and the blood supply is poor. These factors lead to severe soft tissue swelling after ankle fractures. Kadakia et al. [25] revealed that affected by the swelling and pain of the affected area, patients are prone to negative emotions such as tension and anxiety. Results of the study [26] proved about 18% of ankle sprains and up to 23% of ankle fractures will have distal syndesmotic injuries. If the fracture ends are not properly reduced or the joint injury is not clearly diagnosed, serious joint complications can develop over time with a high degree of ankle instability. Benedick et al. [27] mentioned that ankle fracture is an important risk factor for traumatic arthritis. Tension blisters are a common complication of orthopedic surgeons in the treatment of high-energy and low-energy breakages. Due to the lack of soft tissue coverage of the ankle joint and the bony prominence at the joint, tension blisters are prone to form around the fracture end. Commonly seen in the hours following acute injury, blisters are classified into two types: hyperemic and serous, depending on whether the epidermis is completely separated from the dermis [28].

Collins [29] believes that ice packs can constrict local blood vessels, slow down blood circulation, reduce the exudation and swelling of microcirculation and surrounding tissues, and thus achieve the purpose of reducing tissue metabolic rate. The low-temperature environment can also inhibit the inflammatory response and reduce the release of substances such as histamine. The use of cold therapy in the acute phase of fracture can maintain local low temperature, reduce muscle tension, and slow down the conduction velocity of pain nerves, thereby exerting an effective analgesic effect. Lin et al. [30] applied cryotherapy in patients after calcaneal fracture surgery, which can effectively reduce the VAS score, and the infection rate is also greatly reduced. Park et al. [31] believe that in the treatment of limb swelling and pain before ankle fracture surgery, either evaporative coolant with ethanol as the main component or traditional ice packs can achieve good results. Winge et al. [32] are of the view that compression therapy can improve circulation, reduce limb swelling, and prevent it by compressing the circulation of limbs and tissues, promoting the return of blood and lymph, and accelerating the absorption of metabolites, inflammatory factors, and pain-causing factors in the blood. Clarkson et al. [33] mentioned that the use of arteriovenous pneumatic pump therapy after ankle fracture surgery can reduce the swelling of the affected area. Compression cold therapy devices combine cold therapy with air pressure therapy. It is treated according to the set time and temperature. In the acute stage of fracture, the effect of low temperature and pressure can reduce local exudation, constrict blood vessels, improve circulation, and achieve the purpose of relieving pain and controlling inflammation. Application during rehabilitation can prevent joint swelling, reduce muscle soreness, and promote functional recovery of limbs. At the same time, it can effectively avoid the occurrence of adverse events related to cold therapy and give patients a more comfortable experience. It has also been proved that continuous compression and cold therapy within 5 days after ankle arthroscopy can effectively control ankle swelling [34]. In the study [35], patients after total knee arthroplasty were treated with compression and cold therapy for 3 days, and the joint range of motion in the intervention group at discharge was greater than that in the control group.

The concept of dyskinesia is proposed in [36], for the treatment of chronic low back pain. Kinesophobia refers to persistent pain caused by physical activity, which makes the patient have an irrational excessive fear of physical activity, thereby increasing the patient's susceptibility to painful injuries, and even the risk of reinjury. Vlaeyen et al. [37] believe that patients with dyskinesia will show a stronger avoidance behavior to a certain behavior, so it is called the fear-avoidance model. Patients experience cognitive and behavioral changes due to fear of movement. Chung et al. [38] pointed out that fear-avoidance belief is one of the main factors leading to postoperative dysfunction in patients and even generalized pain. Francisco et al. [39] found that fear-avoidance performances may lead to loss of limb function and disability in patients.

## 3. Method

Deep learning (DL) is the emerging domain of machine learning deals with algorithms inspired by the structure and function of the human brain. In this study, a DL approach is utilized for analyzing the rehabilitation effect of patients with orthopedic dyskinesia. Details are presented in the following subsections.

### 3.1. Basic Theory of CNN

The convolutional neural network [40] first uses forward propagation to calculate the output value of the neural network and then updates the weights and biases of the neural network through back propagation. The neurons between adjacent layers in CNN are not fully connected but adopt a sparse connection. In addition to the advantages of traditional artificial neural networks, sparse connections in convolutional neural networks also have regularization effects. This increases the generalization ability of the network, avoids overfitting, and the sparse connection also reduces the number of parameters, reduces computational consumption, and enables the network to learn quickly. In addition, the convolutional neural network can directly use the original data as the input of the network, avoiding the tedious preprocessing operations on the original data and the need for prior knowledge. Generally speaking, a typical convolutional neural network mainly includes operations such as convolutional layers, pooling layers, and fully connected layers. The convolutional layer and the pooling layer cooperate with each other to extract features layer by layer and finally complete the classification through several full connections.

The function of the convolutional layer is to extract features based on the feature map output by the previous layer. The three most significant features of the convolutional layer are local perception, multikernel convolution, and parameter sharing. Each neuron only needs to perceive the local features in the image or feature map, and in the high layer of the network, the network will integrate the local information obtained by the low layer together to obtain a more global information. All neurons in the same layer of the convolutional neural network will share the same set of parameters, so the parameters in each neuron and its corresponding local receptive field will be regarded as a position-independent feature extraction method. If only one convolution kernel is included in the convolutional layer, such feature extraction is obviously insufficient. Therefore, each convolutional layer in the convolutional neural network will use multiple convolution kernels to learn more abundant features. More specifically, the essence of the convolution layer is to calculate a new feature map, and the process is to convolve the input feature map with a learnable convolution kernel. The convolution is to do the inner product of the local receptive field and the convolution kernel, that is, multiply each corresponding element one by one and then sum:

(1) $$\begin{array}{c} f_{k}^{C}=\underset{c}{\sum }\underset{x,y}{\sum }i_{c}\left(x,y\right)e_{k}\left(p,q\right). \end{array}$$

In theory, the local perception and weight sharing mechanism of CNN reduces the complexity and number of parameters of the neural network to a certain extent. But it is still difficult to directly use all the features extracted by the convolution to train the classifier, because the dimension of the features is still very high, and it will lead to the occurrence of overfitting. In order to solve this problem, the pooling layer is used in the convolutional neural network to downsample the feature map, and the structures of different positions are aggregated and counted to achieve the purpose of reducing the dimension of the feature map. In the compression of data, common pooling layers have two forms, namely, max pooling and average pooling. Max pooling selects the maximum value in the local receptive field as its output, while average pooling calculates the average value in the local receptive field as the output:

(2) $$\begin{array}{c} Z_{k}^{C}=g_{p}\left(F_{k}^{C}\right). \end{array}$$

The convolution and pooling operations are both linear transformations, and the linear model is not expressive enough. It is feasible to operate only some linearly separable data. The activation function introduces nonlinear factors, which can divide the data into smooth curves. Approaching a smooth curve can handle various complex nonlinear data more easily, and the neural network also has better expressive ability and can better fit the objective function. Therefore, the activation function, as a decision function, helps to learn a complex model. Choosing an appropriate activation function can speed up the learning process:

(3) $$\begin{array}{c} T_{k}^{C}=g_{a}\left(F_{k}^{C}\right). \end{array}$$

In a fully connected layer, all neurons between adjacent layers are fully connected. The number of input neurons in the fully connected layer is equal to the feature dimension extracted above, the number of output neurons is the same as the number of output categories, and the number of layers and neurons in the hidden layer are designed according to requirements. Furthermore, the output of a convolutional or pooling layer in a convolutional neural network is a multidimensional feature map. Before inputting these multidimensional feature maps to the fully connected layer, all elements of the feature map need to be flattened and concatenated into a one-dimensional vector, which can then be input to the fully connected layer for further computation.

In deep networks, the input data has been artificially normalized. With the step-by-step transmission of input data in each subsequent layer, the distribution of the input data in each subsequent layer will inevitably change, and the problem of internal covariance shift will occur. Batch normalization is used to solve related problems:

(4) $$\begin{array}{c} N_{k}^{C}=\frac{F_{k}^{C}-\mu_{B}}{\sqrt{\mu_{B}^{2}+\varepsilon }},\\ {BN}_{k}^{C}=\gamma N_{k}^{C}+\beta . \end{array}$$

### 3.2. Postoperative Rehabilitation Evaluation with 1D-DenseNet

This paper recommends a deep convolutional neural network based on one-dimensional DenseNet for automatic feature extraction and classification of rehabilitation data.  Figure 1 depicts the overall architecture of the proposed network. The proposed network structure is collected of three dense blocks and transition blocks in the interval. The input of the network is the patient's physiological data, and the network outputs the efficacy evaluation results.

### 3.3. Dense Block

Depending on the complexity of data, there might be multiple convolutional layers in a neural network. For instance, in AlexNet there are only 5 convolutional layers, in VGG there are 19 layers, while in ResNet there are more than 100 layers. In GoogLeNet, different sizes of convolution kernels are used in the inception module to calculate feature maps. A very significant trend in the field of convolutional neural networks is that the current network is becoming deeper and wider, that is, the number of layers stacked in the network is increasing, and the number of parallel layers is increasing. However, simply increasing the depth and width does not actually make much of a difference. It will also bring a large number of parameters to increase the computational burden and bring about problems such as gradient disappearance and gradient explosion. This makes the network very difficult to train and prone to overfitting, which is not applicable in practical applications. In some deep convolutional neural networks in recent years, some new connection methods have been proposed. Recently, a new connection method has been proposed in dense convolutional neural networks (DenseNet) and has shown outstanding results in the field of image recognition. It densely connects the feature maps in each dense module, that is, the output feature map of the previous layer in a module is used as the input of each subsequent layer, and the network becomes simplified by feature reuse. Therefore, this work introduces this connection method into the evaluation of postoperative curative effect of self-made compression cold therapy on orthopedic patients, so as to reduce the parameter consumption of neural network and realize a very simplified neural network method.  Figure 2 shows the structure of a dense block.  Figure 3 illustrates the structure of composite layer.

All feature maps densely connected within a dense module can be viewed as a global state. This not only brings feature reuse capability so that higher layers can directly use the feature maps of lower layers but also enables gradients to be passed more directly to lower layers during backpropagation. In the dense module, this paper selects a composite layer composed of multiple nonlinear operations and uses all the feature maps before this layer as input to calculate the output feature map of this layer. And set the growth rate hyperparameter to control the number of output feature maps of each layer. Although by controlling the growth rate, each composite layer produces only k output feature maps. However, the dimension of the input feature map is still very huge relative to the later layers, so a bottleneck structure composed of operations such as point-by-point convolution is used to control the upper limit of the input dimension. Weight sharing feature is also a feasible approach to reduce the number of trainable parameters and to improve the classification effect of neural network.

### 3.4. Transition Module

If all layers in the network are directly associated in a densely connected manner, the connections in the network will increase squarely. Such a connection pair has a very high consumption of computer memory/memory. If there are *L* layers in the network, there will be *L*(*L* + 1)/2 connections between layers. Therefore, the entire network is split into a way of stacking multiple dense modules, and transition modules are used for spacing between adjacent dense modules. In order to reduce the size of the feature map, the number of trainable network parameters need to be reduced. To improve classification effect, to reduce the training parameters, and to extract more global features, average pooling layer is used in the transition module. In addition, a lightweight interchannel attention mechanism from SENet is introduced into each transition module to achieve weighting between feature map channels. Through learning, the weights of more descriptive structures are increased and the weights of irrelevant features are reduced to ensure that more useful information can be sent to subsequent layers for further feature extraction. The structure of transition module is illustrated in Figure 4.

Specifically, this attention mechanism can be separated into two steps of compression and activation. In the first step, global average pooling is used to compress the information in the spatial dimension of the feature map into a channel description vector whose length is the same as the number of channels of the feature map. This can overcome the problem that the useful context information outside the receptive field cannot be utilized because the convolutional receptive field is too small.

### 3.5. Separable Convolution

Inspired by the construction of lightweight neural networks suggested in Xception and MobileNet [41], the concept of separating correlations between channels and spatial dimensions is utilized in feature maps. The paper announces the separable convolution (SepConv) structure combined with one-dimensional convolution and applies it to the proposed network. Separable convolution mainly separates ordinary convolution into two independent convolutions: channel-independent convolution and pointwise convolution. Definition of pointwise convolution, channel-independent convolution and separable convolution:

(5) $$\begin{array}{c} \text{PointConv}{\left(W,y\right)}_{\left(i\right)}=\overset{C}{\underset{c=1}{\sum }}W_{c}∙y_{\left(i,c\right)},\\ \text{DepthConv}{\left(W,y\right)}_{\left(i\right)}=\overset{K}{\underset{k=-K}{\sum }}W_{k}*y_{\left(i,k\right)},\\ \text{SepConv}{\left(W_{p},W_{d},y\right)}_{\left(i\right)}={\text{DepthConv}}_{\left(i\right)}\left(W_{p},{\text{DepthConv}}_{\left(i\right)}\left(W_{d},y\right)\right). \end{array}$$

It has been proved that correlation between channels and spatial dimensions in the feature map can be completely decoupled [42]. Thus, separating ordinary convolutions can significantly reduce parameters and training time. By this way, the nonlinear ability of the network can be improved. Therefore, in the proposed method, the separable convolution is applied to the dense module instead of the ordinary convolution structure. Compared with the previous network using separable convolution, this method eliminates the residual connection and applies the dense connection method to make the information flow in the network more efficient while using a fewer parameters.

### 3.6. Loss Function

A common problem faced by deep learning models is class imbalance, where some classes have significantly more training samples while others have fewer samples. This usually makes the model tend to choose a large number of categories, but often categories with a small number of samples are more critical for research. The class imbalance problem has significant adverse effects on both convergence in training and generalization in testing. The current existing approaches to address this problem can be divided into two broad categories, namely, data-based methods and classifier-based methods.

In this paper, a classifier-based method is adopted, that is, a weighted cross-entropy loss (WCE) is used as the loss function of this neural network. It is a simple extension of the cross-entropy loss function:

(6) $$\begin{array}{c} \text{WCE}\left(p_{t}\right)=-\alpha_{t}\log\left(p_{t}\right). \end{array}$$

### 3.7. Network Details

The one-dimensional DenseNet deep convolutional neural network proposed in the paper has a total of 44 layers, which can be mainly divided into three dense modules and spaced transition modules, and the number of layers in each dense module is the same. Feature maps before being fed into the first dense module, a large convolutional kernel of size 7 and stride 2 is used to extract low-level features from the input heart sound segments, and a 24-channel feature map is generated. Then, a max pooling of size 3 and stride 2 is used to reduce the size of the feature maps. In this neural network, each dense module contains 6 composite layers, and the growth rate k is set to 12. A smaller kernel is used in all separable convolutions of each dense module, the kernel size is set to 3, and the stride is set to 1. The transition modules of densely spaced modules mainly include pointwise convolution, attention mechanism, and an average pooling of size 2. After the last dense module, a global average pooling is used to convert the feature map into a vector, and full connections and Softmax are used for final classification. See Table 1 for more detailed network structure details about the proposed 1D-DenseNet.

## 4. Experiment and Discussion

This study intends to evaluate efficacy of patients by conducting a comparative study. Details about the dataset and the results obtained from multiple perspectives are given as follows.

### 4.1. Used Dataset

This work uses a self-made dataset to evaluate the efficacy of self-made compression cold therapy in the treatment of dyskinesia in patients undergoing orthopedic surgery. This dataset contains a total of 35,938 samples, of which 23,959 samples are training sets and the remaining 11,979 samples are test sets. The input of each sample is the collected medical data, and the labels correspond to the efficacy grades, which are divided into four different effects. This work is a classification task, and the evaluation metrics used are precision and recall.

### 4.2. Method Comparison

To verify the correctness and effectiveness of the 1D-DenseNet network proposed in this work for evaluating the efficacy of patients, a comparative experiment was conducted. The compared methods include SVM, BP, and 1D-CNN, and the experimental results are shown in Table 2.

It is obvious that the method proposed in this work achieves the highest performance: 96.7% precision and 93.9% recall. Compared to the best strategy of 1D-CNN, 1D-DenseNet can obtain 3.2% precision improvement and 2.1% recall improvement. This verifies the validity and correctness of this work.

### 4.3. Result of Dense Block

As mentioned earlier, this work adopts the dense block strategy. To verify the effectiveness of using this strategy, this work conducts comparative experiments to compare the efficacy evaluation performance with and without dense block, respectively. The experimental results are illustrated in Figure 5.

It is obvious that the highest evaluation performance can be obtained using the dense block. Compared to not using this strategy, 2.1% precision improvement and 1.4% recall improvement can be obtained with a dense block. This verifies the correctness and reliability of the dense block strategy used in this work.

### 4.4. Result of Transition Module

As mentioned earlier, this work adopts the transition module strategy. To verify the effectiveness of using this strategy, this work conducts comparative experiments to compare the efficacy evaluation performance with and without transition module, respectively. The experimental results are illustrated in Figure 6.

It is obvious that the highest evaluation performance can be obtained using the transition module. Unlike other strategies, 1.5% precision improvement and 1.1% recall improvement are achievable with the transition module. This verifies the correctness and reliability of the transition module strategy used in this work.

### 4.5. Result of WCE Loss

As mentioned earlier, this work adopts the WCE loss strategy. To verify the effectiveness of using this strategy, this work conducts comparative experiments to compare the efficacy evaluation performance with and without WCE loss, respectively. The experimental results are illustrated in Figure 7.

It is obvious that the highest evaluation performance can be obtained using the WCE loss. Compared to not using this strategy, 2.3% precision improvement and 2.0% recall improvement can be obtained with a WCE loss. This verifies the correctness and reliability of the WCE loss strategy used in this work.

### 4.6. Result of Attention

As mentioned earlier, this work adopts the attention strategy. To verify the effectiveness of using this strategy, this work conducts comparative experiments to compare the efficacy evaluation performance with and without attention, respectively. The experimental results are illustrated in Table 3.

It is obvious that the highest evaluation performance can be obtained using the attention mechanism. Encouraging results are obtained by comparing results of the proposed method with those which are without the attention mechanism. As a whole, 1.8% precision improvement and 1.2% recall improvement were obtained with the attention mechanism. This verifies the correctness and reliability of the attention mechanism used in this work.

## 5. Conclusion

Due to the particularity of structure and function, ankle fractures are the most common joint fractures in clinical practice. With the enrichment of leisure life and the development of social aging, the incidence rate has also increased. Surgery is an effective way to treat ankle fractures. The existence of surgical incisions may main to tissue nerve damage, soft tissue swelling, and pain. If these problems cannot be solved in a timely and effective manner, various complications will occur. Most patients have postoperative kinesiophobia due to pain, and compression cold therapy can control refrigeration and reduce the possibility of tissue damage. Therefore, it is very important to evaluate the efficacy of self-made compression cold therapy on patients with dyskinesia after orthopedic surgery. This will help the medical staff to formulate the next treatment plan. This work proposes a one-dimensional deep convolutional neural network-based technique for analyzing the rehabilitation effect of patients with kinesiophobia after ankle fracture surgery. This work proposes a one-dimensional DenseNet-based network to evaluate the rehabilitation effect of self-made compression cold therapy on patients with orthopedic dyskinesia. In this paper, a deep convolutional neural network with low parameter consumption is constructed starting from the feature reuse of convolutional neural network, attention mechanism, correlation decomposition of feature map space, and channel dimension. Comprehensive and systematic experiments verify the correctness and efficiency of this work. In the future, we are determined to utilize the proposed approach in evaluating efficacy of the surgical treatment of knee arthroplasty, a rising resurfacing surgical technique.

## Figures and Tables

**Figure 1:** The structure of 1D-DenseNet.

**Figure 2:** The structure of dense block.

**Figure 3:** The structure of composite layer.

**Figure 4:** The structure of transition module.

**Figure 5:** Result of dense block.

**Figure 6:** Result of transition module.

**Figure 7:** Result of WCE loss.

**Table 1:** Detailed structure configuration.

Layer	Output size	Configuration
Conv	1 × 2500 × 24	Conv 1 × 7
Pool	1 × 1250 × 24	Maxpool 1 × 3
Dense block (1)	1 × 1250 × 96	Composite layer *k* = 12
		SepConv 1 × 3
Transition module (1)	1 × 625 × 48	PointConv
		Attention
		Avgpool 1 × 2
Dense block (2)	1 × 625 × 120	Composite layer *k* = 12
		SepConv 1 × 3
Transition module (2)	1 × 312 × 60	PointConv
		Attention
		Avgpool 1 × 2
Dense block (3)	1 × 312 × 120	Composite layer *k* = 6
		SepConv 1 × 3
Classifier	1 × 1 × 120	GAP
	4	FC

**Table 2:** Comparison between different methods.

Method	Precision	Recall
SVM	87.90	85.61
BP	91.20	88.71
1D-CNN	93.50	91.81
1D-DenseNet	96.70	93.91

**Table 3:** Result of attention mechanism.

Method	Precision	Recall
No attention	94.9	92.7
Have attention	96.7	93.9

## Data Availability

The datasets used during the current study are available from the corresponding author on reasonable request.
